# Application Effect of Medical Care Integration Combined with Family Intervention under the Evidence-Based Nursing Mode on Child Patients with Severe Hand-Foot-Mouth Disease and Its Influence on Intestinal Function

This article has been retracted.

**DOI:** 10.1155/2021/9599711

**Published:** 2021-10-11

**Authors:** Zhaofang Zhang, Mei Dong, Yuejiao Han, Hui Lin, Anying Li, Na Wang, Xia Zhang

**Affiliations:** ^1^Department of Nursing, Qilu Children's Hospital of Shandong University, Jinan 250022, Shandong Province, China; ^2^Operation Room, Shandong Provincial Hospital, Jinan 250021, Shandong Province, China; ^3^Department of Neonatology, Qilu Children's Hospital of Shandong University, Jinan 250022, Shandong Province, China; ^4^Department of Calm Center, Qilu Children's Hospital of Shandong University, Jinan 250022, Shandong Province, China; ^5^Department of Infectious, Qilu Children's Hospital of Shandong University, Jinan 250022, Shandong Province, China; ^6^Endoscopy Room, The Fourth People's Hospital of Jinan, The Third Affiliated Hospital of Shandong First Medical University, Jinan 250031, Shandong Province, China

## Abstract

**Objective:**

To explore the application effect of medical care integration combined with family intervention under the evidence-based nursing mode on child patients with severe hand-foot-mouth disease (HFMD) and its influence on intestinal function.

**Methods:**

120 child patients with severe HFMD admitted to Qilu Children's Hospital of Shandong University from January 2019 to January 2020 were selected as the research object and randomly divided into group A and group B, with 60 cases each. Conventional nursing was performed on patients in group B, and medical care integration combined with family intervention under the evidence-based nursing mode was performed on patients in group A. Patients were assessed after the intervention using the hospital-made treatment adherence scale, PedsQLTM 4.0 (Pediatric Quality of Life Inventory Version 4.0) scale, and the faces pain scale-revised (FPS-R). The levels of gastrointestinal function indicators such as serum endotoxin (ET), diamine oxidase (DAO), and d-lactic acid (D-LA) were measured before and after the intervention, and recovery such as time to clear fever and time to relief of oral pain were recorded in both groups.

**Results:**

Children in group A had significantly higher compliance in diet, behaviour, exercise, and medication than group B (*P* < 0.05); the time to clear fever, time to relief of oral pain, time to healing of oral ulcers, time to relief of skin herpes, time to hospitalization, and time to eating were shorter in group A than those in group B (*P* < 0.001); all scores on the PedsQLTM 4.0 scale were higher in group A than those in group B after the intervention (*P* < 0.001); ET, DAO, and D-LA levels decreased in both groups after the intervention, with group A having lower levels than group B (*P* < 0.001), in addition, group A had lower eating pain scores after the intervention (*P* < 0.05).

**Conclusion:**

Medical care integration combined with family intervention under the evidence-based nursing mode can effectively improve the treatment compliance of child patients with severe HFMD, accelerate their recovery progress, ensure a better prognostic quality of life and gastrointestinal tract function, and reduce the eating pain, indicating that such comprehensive nursing intervention mode should be promoted in practice.

## 1. Introduction

Hand-foot-mouth disease (HFMD) is mostly caused by enterovirus (EV) infection, so children with HFMD usually present with impaired intestinal function, and in the exacerbation phase, the symptoms such as fever and rash become more severe and some children experience intense pain, which significantly affect their daily life in an adverse way [1–3]. As children with HFMD are young and their treatment adherence is low, the usual care model adopted in the clinic is less effective in improving the outcomes of critically ill children with HFMD, so there is no time to delay in changing the care model. In recent years, with the increasing awareness of the discipline of nursing, the health-care integration treatment mode is gradually being applied in practice, which aims to change the subordinate status of nursing personnel so that they can perfect the treatment and nursing together with the clinicians, thereby improving the efficiency and quality of clinical care and enhancing the rehabilitation effect of patients [4–7]. For critically ill children with HFMD who have a poor prognosis, the application of a health-care integration mode is essential, during which nursing personnel can deepen their understanding of HFMD with the help of evidence-based care and then provide better-quality care services to children. In addition, critically ill children are at higher risk of developing complications such as pulmonary edema, meningitis, or circulatory failure and require strict clinical care [8–11]. From evidence-based data, performing family care while receiving hospital care can reduce the likelihood of complications and improve overall survival chances of children. Family care refers to therapeutic care, medication care, and visiting care from family members, and good family care is the key to improving the recovery of children. To explore the application effect of medical care integration combined with family intervention under the evidence-based nursing mode on critically ill children with HFMD and its influence on gastrointestinal tract function, 120 critically ill children with HFMD admitted to our hospital from January 2019 to January 2020 were selected for the study, with the results summarized as follows.

## 2. Materials and Methods

### 2.1. General Information

A total of 120 critically ill children with HFMD admitted to Qilu Children's Hospital of Shandong University from January 2019 to January 2020 were selected as the research object and randomly divided into group A and group B, with 60 cases each. No statistical differences were presented when comparing the child patients' general information between the two groups (*P* > 0.05); see Table 1. The study was approved by the hospital ethics committee.

### 2.2. Inclusion Criteria

The inclusion criteria of the study were as follows. (1) The family members of the children fully understood the study process and signed the informed consent; (2) the children were diagnosed with severe HFMD after examination according to the 2010 version of *Diagnosis and Treatment Guidelines for Hand-foot-mouth Disease* [12]; and (3) the children had the fever symptom [13].

### 2.3. Exclusion Criteria

The exclusion criteria for child patients of the study were as follows. (1) Presence of mental problems or inability to communicate with others; (2) suffering from other organic diseases; (3) under coma [14]; (4) with combined hereditary diseases or the presence of brain injury [15]; and (5) presence of prior epilepsy history and other diseases.

### 2.4. Methods

Conventional nursing was performed on patients in group B, namely, giving relevant health guidance to the parents of the children for them to memorize the key points of daily care and, at the same time, conducting medication intervention and mental intervention according to condition of the children and providing a good and well-disinfected convalescent environment.

Medical care integration combined with family intervention under the evidence-based nursing mode was performed on patients in group A with the following steps. (1) A medical care integration evidence-based nursing group was established, with the members being allocated according to their seniority, working competence, and other aspects, which was consistent with the allocation of group B; members of the group should establish the medical care integration and intervention log to comprehensively record the disease information, assay information, and appointment time of child patients, as well as their medical care intervention plan and execution status, so as to follow-up their recovery progress in detail. (2) Members of the group should go through relevant literature about severe HFMD, prepare corresponding nursing handbooks for child patients in combination of clinical treatment and nursing experience, and dispense the handbooks to the family members of the child patients in group A and then hold special lectures for the family members to fully learn the specific matters in the nursing handbook, especially the methods of observing the disease, thereby enhancing their ability of identifying the complications and improving the quality of family intervention. (3) Members of the group should adopt the medical-nursing integration ward inspection mode and conduct ward inspection twice per day to learn the changes in the children's condition and adjust the intervention plan in combination with the evidence-based data; during ward inspection, the nursing personnel and doctors should pay attention to the execution of child patients' diet plan and exercise plan and, by fully learning the mental intervention methods in the evidence-based information, grasp their potential mental problems and observe their daily mental change; in case of the presence of poor mental status, the adverse effect on child patients from treatment and nursing should be reduced and the physical touch with the child patients should be increased to promote their sense of trust. (4) Members of the group should make intervention decisions according to the demands of child patients' family members, so as to enhance their nursing confidence and increase the nursing compliance of child patients; after the discharge of child patients, members of the group conducted regular follow-up visits to ask their family members about the implementation of the family intervention program, and monthly HFMD knowledge reviews were held to ensure that their family members had adequate awareness of the condition.

### 2.5. Observation Criteria

1. Treatment compliance: after the nursing intervention, the adherence to treatment of the paediatric patients was evaluated and compared according to a questionnaire proposed by our hospital, with items including diet, medication, exercise, and behaviour. If the children fully obeyed the medical advice, it was regarded as good compliance, and in the case of being reluctant to follow the medical advice, following the medical advice passively, or failure to follow the medical advice at all, it was regarded as poor compliance.
2. Recovery-related indexes: time to clear fever, time of oral pain alleviated, time of oral ulcer healed, time of skin herpes alleviated, length of stay [16], and feeding time were observed and recorded in both groups of children, and the results were collated and compared.
3. Quality of life: after the nursing intervention, the PedsQLTM 4.0 (Pediatric Quality of Life Inventory Version 4.0) scale was used as the basis to evaluate the quality of life of children after intervention, corresponding items were selected for evaluation according to the age group of children, and those without the evaluation ability were completed by their family members. The evaluation items included physical, character, emotional, and social functions, and the maximum score of each item was 100 points, with higher scores indicating better condition of children [17, 18].
4. Gastrointestinal tract function indexes: 3 mL of fasting venous blood was collected from all children before and after the intervention, and the serum was centrifuged and stored in a refrigerator at −80°C. The levels of serum endotoxin (ET), diamine oxidase (DAO), and d-lactic acid (D-LA), which are markers of gastrointestinal function, were measured in both groups using an enzyme-linked immunoassay kit, and the results were recorded and collated.
5. Eating pain scores: after the intervention, the eating pain sense of children was evaluated according to the faces pain scale-revised (FPS-R) on a scale of 0–10 points, with 2 points and below indicating mild pain, 3 points indicating moderate pain, and 4 points and above indicating severe pain, so as to compare their pain scores [19].

### 2.6. Statistical Processing

In this study, the data processing software was SPSS20.0, and the picture drawing software was GraphPad Prism 7 (GraphPad Software, San Diego, USA). The measurement data are expressed as mean ± standard deviation (Mean ± SD) using the *t*-test; the count data are expressed as cases (*n*) using the X^2^ test and rank data using the rank sum (*z*) test. Also, differences were considered statistically significant at *P* < 0.05.

## 3. Results

### 3.1. Comparison of Children's Treatment Compliance

The treatment compliance of group A was significantly higher than that of group B (*P* < 0.05); see Figure 1.

Compared with group B, group A had significantly higher number of children with diet compliance (58 cases vs. 45 cases, *P* < 0.05), behavior compliance (54 cases vs. 45 cases, *P* < 0.05), exercise compliance (58 cases vs. 48 cases, *P* < 0.05), and medication compliance (54 cases vs. 42 cases, *P* < 0.05).

### 3.2. Comparison of Children's Recovery-Related Indexes

Group A obtained significantly better recovery-related indexes than group B (*P* < 0.001); see Table 2.

### 3.3. Comparison of Children's Quality of Life

Group A presented significantly better quality of life than group B after intervention (*P* < 0.001); see Table 3.

### 3.4. Comparison of Children's Gastrointestinal Tract Function Indexes

After intervention, the gastrointestinal tract function of children in group A was significantly better than that of children in group B (*P* < 0.001); see Table 4.

### 3.5. Comparison of Children's Eating Pain Scores

The eating pain scores were significantly lower in group A than those in group B (*P* < 0.05); see Figure 2.

Respectively, the numbers of cases with eating pain scores of ≤2 points, 3 points, and ≥4 points in group A were significantly smaller than those in group B (12 cases vs. 4 cases, *P* < 0.05; 45 cases vs. 34 cases, *P* < 0.05; and 3 cases vs. 22 cases, *P* < 0.05).

## 4. Discussion

HFMD is a common clinical condition mostly caused by EV infection, and children with the disease usually develop a skin rash at the end of the hands and feet, and some even have oral ulcers, fever, and other clinical symptoms, which seriously affect their daily life. Although a large proportion of children with HFMD are less symptomatic and can recover after systematic therapeutic intervention, some who develop into severe HFMD with extremely rapid progression have a higher likelihood of developing complications such as pulmonary edema and meningitis, and the risk of death is substantially higher if no interventional therapeutic intervention is performed [20–22].

Complications are the key in influencing outcomes of critically ill children with HFMD, so nursing personnel have shifted the clinical nursing mode and applied the evidence-based nursing in the care of children with HFMD. By reviewing the literature and combining with their own experience, nursing personnel can fully grasp the risk factors in the care of critically ill children with HFMD and improve their ability to identify risk factors, and at the same time, combined with part of the evidence-based data, it is reasonable to adopt the family nursing intervention while performing hospital nursing intervention to enable the children to receive dual care, thereby comprehensively reducing the likelihood of developing complications and optimizing recovery in affected children. For critically ill children with HFMD, the simultaneous acquisition of multiple care models under the guidance of evidence-based care is the key to improve their outcomes. Nowadays, with the increasing emphasis on nursing, health-care integration intervention has become a popular direction of clinical research, which can improve the collaborative efficiency of doctors and nursing personnel, so that children receive comprehensive intervention with better quality. Therefore, the rehabilitation-related indexes (*P* < 0.001) and improvement in gastrointestinal function (*P* < 0.001) obtained in group A were significantly better than those in group B. This indicates that such integrated medical care mode could effectively accelerate the recovery process of critically ill children with HFMD and had higher clinical application value.

In addition, the results of the study also showed that the compliance of children in group A in terms of diet, behavior, exercise, and medication (*P* < 0.05) and the scores of the PedsQLTM 4.0 scale after intervention (*P* < 0.001) were significantly higher than those in group B. Children with severe HFMD are usually less tolerant and more resistant to treatment and have low treatment compliance that tends to be reduced again after discharge from hospital, which is detrimental to their body rehabilitation [23, 24]. In this study, the families of children in group A were educated on the knowledge of HFMD, aiming to improve the family nursing intervention ability of their family members and enhance the awareness of the identification of risk factors, so the children in this group still received efficient care after discharge from hospital, kept a better treatment compliance, and obtained a more rapid rehabilitation, which ensured a better quality of life for them.

The research of Priyia et al. [25] and others presented that feeding time and eating pain scores could be used as the important indicators for evaluating the prognosis of critically ill children with HFMD, and this study showed that group A had significantly lower feeding time (*P* < 0.001) and eating pain scores (*P* < 0.05) than group B after intervention, which was consistent with the finding of Priyia et al. In their research, dual nursing of hospital and family was performed on children in the experimental group, and hospital nursing was conducted for children in the control group, and it was concluded that the eating pain scores after intervention were significantly lower in the experimental group than in the control group (*P* < 0.001), indicating that the nursing mode combining hospital nursing with family nursing was more conducive to the recovery of critically ill children with HFMD.

In conclusion, medical care integration combined with family intervention under the evidence-based nursing mode can effectively improve the treatment compliance of child patients with severe HFMD, accelerate their recovery progress, ensure a better prognostic quality of life and gastrointestinal tract function, and reduce the eating pain, indicating that such comprehensive nursing intervention mode should be promoted in practice.

## Figures and Tables

**Figure 1:** Comparison of children's treatment compliance. The horizontal axis from left to right indicates diet compliance, behavior compliance, exercise compliance, and medication compliance, and the vertical axis indicates children (cases); the black areas indicate group A, and the gray areas indicate group B; ^*∗*^ indicates *P* < 0.05.

**Figure 2:** Comparison of children's eating pain scores. The horizontal axis from left to right indicates ≤2 points, 3 points, and ≥4 points, and the vertical axis indicates children (cases); the black areas indicate group A, and the gray areas indicate group B; ^*∗*^ indicates *P* < 0.05.

**Table 1:** Comparison of child patients' general information.

Group	Group A (*n* = 60)	Group B (*n* = 60)	*X* ^2^/*t*/*z*	*P*
Gender (*n*)			0.033	0.855
Male	30	31		
Female	30	29		
Mean body temperature (°C, mean ± SD)	38.98 ± 0.21	38.95 ± 0.23	0.746	0.457
Mean age (years, mean ± SD)	5.40 ± 1.21	5.41 ± 0.91	0.051	0.959
HFMD symptom (*n*)				
Drooling	45	46	0.046	0.831
Food refusal	35	34	0.034	0.853
Dysthesia	32	31	0.033	0.855
Oral burning sensation (*n*)	42	40	0.154	0.695
Buttock rash (*n*)	36	37	0.035	0.852
Rash at the end of the hands and feet (*n*)	55	56	0.120	0.729
Convulsion (*n*)	20	23	0.326	0.568
Mean disease duration (*d*, mean ± SD)	3.54 ± 0.54	3.56 ± 0.37	0.237	0.813
Appearance time of mouth herpes (*d*, mean ± SD)	1.29 ± 0.21	1.28 ± 0.22	0.255	0.799
Education degree of parents (*n*)			−0.218	0.827
Senior high school and below	17	14		
Junior college/university	38	40		
Above university	5	6		

**Table 2:** Comparison of children's recovery-related indexes (mean ± SD, *d*).

Group	Fever clearance time	Time of oral pain alleviated	Time of oral ulcer healed	Time of skin herpes alleviated	Length of stay	Feeding time
Group A (*n* = 60)	2.78 ± 0.21	2.12 ± 0.20	2.89 ± 0.75	3.45 ± 0.35	7.54 ± 0.87	4.10 ± 0.35
Group B (*n* = 60)	4.25 ± 0.35	3.10 ± 0.68	3.68 ± 0.70	5.48 ± 0.42	8.87 ± 1.10	6.24 ± 0.31
*t*	27.897	10.710	5.965	28.761	7.346	35.454
*P*	<0.001	<0.001	<0.001	<0.001	<0.001	<0.001

**Table 3:** Comparison of children's quality of life after intervention (mean ± SD, points).

Group	Physical score	Character score	Emotional score	Social score
Group A (*n* = 60)	70.11 ± 4.98	66.98 ± 5.48	72.68 ± 5.98	69.98 ± 5.44
Group B (*n* = 60)	58.98 ± 5.98	54.12 ± 5.65	62.11 ± 5.74	54.87 ± 4.58
*t*	11.078	12.656	9.877	16.459
*P*	<0.001	<0.001	<0.001	<0.001

**Table 4:** Comparison of children's gastrointestinal tract function indexes (mean ± SD).

Group	ET (EU/ml)		DAO (U/ml)		D-LA (mg/L)	
	Before intervention	After intervention	Before intervention	After intervention	Before intervention	After intervention
Group A (*n* = 60)	0.65 ± 0.11	0.43 ± 0.05	7.40 ± 0.68	3.65 ± 0.45	14.98 ± 1.98	8.11 ± 1.23
Group B (*n* = 60)	0.66 ± 0.12	0.58 ± 0.03	7.41 ± 0.64	4.55 ± 0.65	14.67 ± 1.94	12.32 ± 1.56
*t*	0.476	19.926	0.083	8.818	0.866	16.415
*P*	0.635	<0.001	0.934	<0.001	0.388	<0.001

## Data Availability

The primary data to support the results of this study are available at reasonable request to the corresponding author.
